# Albiflorin Alleviates Ox-LDL-Induced Human Umbilical Vein Endothelial Cell Injury through IRAK1/TAK1 Pathway

**DOI:** 10.1155/2022/6584645

**Published:** 2022-05-13

**Authors:** Yeling Liu, Yilai Sun, Xue Bai, Lingxing Li, Guihua Zhu

**Affiliations:** ^1^Department of Pharmacy, Tai'an City Central Hospital, Tai'an, Shandong 271000, China; ^2^Department of Pancreatic & Hernial Surgery Tai'an City Central Hospital, Tai'an, Shandong 271000, China; ^3^Department of Cardiovascular Medicine, Tai'an City Central Hospital, Tai'an, Shandong 271000, China

## Abstract

**Introduction:**

Atherosclerosis (AS) is a chronic inflammatory disease characterized by lipid metabolism disorder and vascular endothelial damage. Albiflorin (AF) has been certified to be effective in the therapy of certain inflammatory diseases, while the therapeutic effect and mechanism of AF on AS have not been fully elucidated. *Material and Methods*. Model cells for AS were created by inducing oxidized low-density lipoprotein (Ox-LDL) in human umbilical vein endothelial cells (HUVECs). After processing with AF and interleukin-1 receptor-associated kinase 1- (IRAK1-) overexpressed plasmid, cell viability was assessed by CCK-8; cholesterol efflux was tested using liquid scintillation counter; IL-6 and TNF-*α* levels were determined with ELISA kits; ROS and apoptosis were confirmed using Flow cytometry. Besides, IRAK1-TAK1 pathway and apoptosis- and mitochondrial fusion-related proteins were monitored with western blotting analysis.

**Results:**

Our results verified that AF could not only dramatically accelerate viability and cholesterol efflux but also attenuate inflammation, ROS production, and apoptosis in Ox-LDL-induced HUVECs. Meanwhile, AF could prominently prevent the activation of IRAK1-TAK1 pathway, downregulate apoptosis-related proteins, and upregulate mitochondrial fusion-related proteins in Ox-LDL-induced HUVECs. Moreover, we testified that IRAK1 overexpression memorably could reverse suppression of AF on inflammation, apoptosis, and IRAK1-TAK1 pathway and enhancement of AF on viability, cholesterol efflux, and mitochondrial fusion in Ox-LDL-induced HUVECs.

**Conclusions:**

By blocking the IRAK1/TAK1 pathway, AF can significantly slow the course of AS, suggesting that it could be a viable therapeutic option for AS.

## 1. Introduction

Cardiovascular disease (CVD) is the leading cause of death worldwide, causing about 17.3 million deaths each year [1]. The main pathological process of CVD is atherosclerosis (AS) [2]. AS is a chronic, progressive disease that is characterized by cell activation, lipid infiltration, thrombosis, and an inflammatory immunological response that results in the formation of AS plaques on arterial walls [3, 4]. And AS is defined by the buildup of lipids and inflammatory cells in the walls of the major arteries [5]. Currently, the treatment strategies for AS mainly include (1) lipid-lowering strategies (low-fat diet and the application of statin drugs); (2) strict control of cardiovascular risk factors; and (3) the use of antiplatelet agents for complications caused by AS plaque rupture and local thrombosis, such as acute myocardial infarction and cerebral infarction [6–8]. The incidence of cardiovascular events remained high even when optimal treatment was chosen in AS. It is reported that the incidence of new cardiovascular events is as high as 20% in the first three years after the onset of acute coronary syndrome (ACS) [9]. Researches testified that the pathogenesis of AS involves the functional changes of endothelial cells, smooth muscle cells, and macrophages in blood vessels [10, 11]. Endothelial cells, as the main cellular component of the endarterium, can form an anti-inflammatory signaling network to prevent pathogens from overreacting [12]. Therefore, it has become a new direction of current research to further study the mechanism of changes in vascular endothelial cell function in AS and to combine drugs with different mechanisms to achieve the purpose of alleviating AS lesions.

Radix Paeoniae Rubra (RPR) is a traditional Chinese medicine derived from the dried root of Paeonia lactiflora Pall. or Paeonia veitchii Lynch [13]. RPR has a wide range of pharmacological effects, such as eliminating stasis to stop pain, removing heat to cool blood, and protecting liver, antithrombus, and antitumor [14, 15]. RPR contains a mass of monoterpene glycosides, which are considered as the main active components of RPR, especially paeoniflorin and albiflorin (AF) [16]. Radix Paeoniae Alba (RPA) is similar to RPR in origin, and both of them contain vast monoterpene glycosides [17]. Modern pharmacological researches certified that paeoniflorin has a variety of effects, such as analgesia, anti-inflammation, hypoglycemia, antiplatelet aggregation, antithrombus, antioxidation, and anticonvulsion, which mainly acts on the blood system, nervous system, and endocrine system [18–22]. AF is an isomer of paeoniflorin with similar chemical structure. Since AF content is lower than paeoniflorin and it is difficult to isolate and purify, pharmacological effects of AF are less studied. Recent researches testified that AF was relevant to pulmonary inflammation [23], memory deficits [24], and AS [25]. However, the role and mechanism of AF in alleviating AS is still incomplete.

In the current study, we used oxidized low-density lipoprotein (Ox-LDL) to stimulate human umbilical vein endothelial cells to create a cellular model of AS (HUVECs). Then, we explored the influences of AF on the related biological functions (viability, cholesterol efflux, inflammation, ROS, and apoptosis) of AS model cells. Moreover, we revealed the possible mechanisms of AF in alleviating HUVEC injury induced by Ox-LDL. Thus, AF might provide a new therapeutic opportunity for AS treatment.

## 2. Materials and Methods

### 2.1. Cell Culture

HUVECs were provided by American Type Culture Collection (ATCC, Manassas, USA) and maintained in DMEM medium (Gibco, USA; Cat. No. 21063-029) with 10% fetal bovine serum (FBS, HyClone) at 37°C with 5% CO_2_.

### 2.2. Establishment and Treatment of as Model Cells

The cultured HUVECs were stimulated using 100 mg/L Ox-LDL (Shanghai Yeasen Biotechnology Co. Ltd. Shanghai, China) in endothelial basal medium for 24 h, and Ox-LDL-induced HUVECs were treated with 0, 4, 20, 100, 200, and 300 *μ*M AF for 24 h, respectively. Vector (control) and IRAK1-overexpressed plasmids were purchased from Origene (Rockville, MD, USA). Ox-LDL-induced HUVECs were evenly placed into a 6-well plate and cultured for 12 h at 37°C. Then, the cells were transfected with the vector and IRAK1-overexpressing plasmid with Lipofectamine 3000 (Invitrogen, Waltham, MA, USA) on the basis of the instructions.

### 2.3. CCK-8 Assay

HUVECs were inoculated uniformly into 96-well plates at a rate of 1 × 10^4^/well. The HUVECs were treated based on the experimental purpose, respectively, and each group had 6 duplicate holes. After routine culture for 0, 24, 48, and 72 h, HUVECs in each well were added with 10 *μ*L CCK-8 reagent (Dojindo, Japan). After 3 h of culture, the OD value at 450 nm was tested with a microplate analyzer.

### 2.4. Detection of Cholesterol Efflux

As described in previous literature [26], HUVECs were coincubated with proper amount of cholesterol and medium containing 10%FBS for 48 h. Then, the cells were washed twice with PBS, and HUVECs in each group were treated separately based on the purpose of the study. The treated HUVECs were incubated in the medium containing 0.3%BSA for 48 h and in the medium containing 10 mg/L ApoAI without FBS for another 12 h. Cholesterol in cell supernatants, and the cells was determined by scintillation counting. Cholesterol efflux = [CPM of culture medium/(CPM value of culture medium + CPM of cells)] × 100%(CPM is the count per minute).

### 2.5. ELISA Assay

On the basis of the instructions, IL-6 and TNF-*α* levels were verified using IL-6 ELISA kit (eBioscience, CA, USA) and TNF-*α* ELISA kit (eBioscience, CA, USA), respectively [27].

### 2.6. Flow Cytometry for Apoptosis

The HUVECs were evenly inoculated into 6-well plates at a rate of 5 × 10^5^/well. After processing in line with different groups, HUVECs were washed 3 times with precooled PBS. After centrifugation and resuspended, HUVECs were dyed with propidium iodide (PI) and Annexin V-FITC based on the instructions of Annexin V-FITC/PI Apoptosis Detection Kit (Sigma; Cat. No. APOAF-20TST). Cell apoptosis was tested and analyzed using flow cytometry (Becton-Dickinson FACScan).

### 2.7. Flow Cytometry for ROS

The harvested HUVECs (1 × 10^6^ cells/well) in each group were inoculated into a 6-well plate and addressed with 2.5 mmol/L DCFH-DA (Cat. No. d6883) at 37°C for 25 min. After washing and staining, the fluorescence intensity values were detected by flow cytometry.

### 2.8. Western Blot Assay

Total proteins were extracted with RIPA lysate from the collected HUVECs in each group, and protein concentration was tested by BCA method (Beyotime, China). Protein samples (40 *μ*g) were separated by 10% SDS-PAGE and transferred to PVDF membranes (Roche). PVDF membranes were blocked with 5% skimmed milk powder at room temperature for 2 h and incubated with primary antibody (dilution ratio: 1∶1000) overnight at 4°C and secondary antibody (dilution ratio: 1∶2000) at 37°C for 2 h. The membranes were addressed with ECL solution (Thermo Fisher Scientific), and the results were acquired with a gel imaging system. p-IRAK1 is referenced by IRAK1, p-TAK1 is referenced by TAK1, and GAPDH was applied as the reference for the other proteins. Anti-interleukin-1 receptor-associated kinase 1 (IRAK1), anti-p-IRAK1, anti-TGF-beta-activated kinase 1 (TAK1), anti-p-TAK1, anti-Bax, anti-caspase 3, anti-mitofusion1 (MFN1), anti-mitofusion2 (MFN2) and anti-opticatrophy1 (OPA1) were all purchased from Abcam (USA) [28].

### 2.9. Immunofluorescence (IF) Assay

The collected HUVECs (1 × 10^5^ cells/well) in each group were inoculated into sterile cover glasses in a 6-well plate, respectively. After incubation overnight, HUVECs were fixed by 4% paraformaldehyde (Sigma, St. Louis, MO, USA) and permeated by 0.5%Triton X-100. After sealing with normal goat serum, the HUVECs were exposed with anti-p-TAK1 (1 : 50, Abcam, St. Louis, MO, USA) overnight at 4°C and fluorescent secondary antibody (1 : 100; Abcam, St. Louis, MO, USA) at 37°C for 1 h. After DAPI (Thermo Fisher Scientific, Waltham, MA, USA) nucleation, the fluorescence intensity was observed using a fluorescence microscope (Olympus, CKX41) [29].

### 2.10. Statistical Analysis

Statistical analysis was conducted using SPSS 21.0 (SPSS Inc., Chicago, IL, USA); statistical graphs was made using GraphPad Prism 8 software. The experimental data was represented as mean ± SD. One-way analysis of variance (ANOVA) was adopted for data comparison among multiple groups, and *P* < 0.05 was for statistically significant.

## 3. Results

### 3.1. AF Memorably Induced Viability and Cholesterol Efflux and Repressed Inflammation, ROS Production, and Apoptosis in Ox-LDL-Induced HUVECs

To determine the impacts of AF on the related functions of Ox-LDL-induced HUVECs, we adopted different concentration of AF (0, 4, 20, 100, 200, and 300 *μ*M) to stimulate HUVECs. As displayed in Figure 1(a), the inhibition rate of HUVECs was significantly elevated with the increase of AF concentration, and the inhibition rate was the highest in the 300 *μ*M AF group. Then, cellular model of AS was established with HUVECs through stimulation of 100 mg/L Ox-LDL, and model cells were processed with 4 *μ*M and 100 *μ*M AF, which were selected based on the CCK-8 results above. Subsequently, the CCK-8 data signified that cell viability was observably attenuated in Ox-LDL group relative to that in control group, while cell viability was signally enhanced in Ox-LDL+100 *μ*M AF group versus that in Ox-LDL group (Figure 1(b)). Meanwhile, we discovered that Ox-LDL induction could lead to a noteworthy increase in cholesterol efflux, and AF treatment also could further increase the cholesterol efflux in Ox-LDL-induced HUVECs, especially 100 *μ*M AF group (Figure 1(c)). ELISA results denoted that Ox-LDL stimulation could result in a remarkable elevation in IL-6 and TNF-*α* levels, while this elevation also could be notably weakened by AF, especially 100 *μ*M AF in Ox-LDL-induced HUVECs (Figure 1(d)). Besides, the data from flow cytometry represented that the level of ROS in the Ox-LDL group was dramatically higher than the control group, while ROS level was in the Ox-LDL + AF group was significantly lower than the Ox-LDL group (Figure 1(e)). Similarly, the data exhibited that cell apoptosis was prominently potentiated in Ox-LDL group with respect to that in control group, while cell apoptosis was signally attenuated in Ox-LDL+AF group compared to that in Ox-LDL group, especially 100 *μ*M AF group (Figure 1(f)). As a whole, we proved that AF, as a possible therapeutic drug, can affect the viability, cholesterol efflux, inflammation, ROS production, and apoptosis of Ox-LDL-induced HUVECs.

### 3.2. AF Dramatically Suppressed IRAK1-TAK1 and Apoptosis and Induced Mitochondrial Fusion in Ox-LDL-Induced HUVECs

Subsequently, we further illuminated the underlying mechanisms by which AF can improve the functions of Ox-LDL-induced HUVECs. Firstly, western blotting results uncovered that the levels of p-IRAK1 and p-TAK1 were memorably elevated in Ox-LDL group versus that in control group, while this elevation of p-IRAK1 and p-TAK1 expressions mediated by Ox-LDL could be partially reversed by AF in HUVECs, especially 100 *μ*M AF (Figure 2(a)). Secondly, the results revealed that Ox-LDL stimulation dramatically upregulated apoptosis-related proteins (Bax and caspase 3) and downregulated mitochondrial fusion-related proteins (MFN1, MFN2, and OPA1), while Ox-LDL-mediated changes in the expression of these proteins could also be prominently reversed by AF in HUVECs, especially 100 *μ*M AF (Figure 2(b)). Moreover, IF results further verified that Ox-LDL treatment could result in a prominent increase in p-TAK1 expression, while the introduction of AF could notably reverse p-TAK1 expression in Ox-LDL-induced HUVECs, especially 100 *μ*M AF group (Figure 2(c)). On the whole, these findings manifested that AF could dramatically affect apoptosis, mitochondrial fusion, and IRAK1-TAK1 pathway in Ox-LDL-induced HUVECs.

### 3.3. AF Markedly Suppressed Inflammation and Enhanced Viability and Cholesterol Efflux by Inhibiting IRAK1 in Ox-LDL-Induced HUVECs

Based on the above result that AF could prevent IRAK1-TAK1 pathway, we speculated that IRAK1-TAK1 pathway might be involved in the change process of Ox-LDL-induced HUVECs function mediated by AF. In order to further confirm this hypothesis, we conducted a rescue experiment in Ox-LDL-induced HUVECs. Above all, 100 *μ*M AF and IRAK1-overexpressed plasmid were applied to coprocess Ox-LDL-induced HUVECs. CCK-8 data disclosed that overexpression of IRAK1 could observably reverse the enhancement of AF (high doses) on cell viability in Ox-LDL-induced HUVECs (Figure 3(a)). Simultaneously, ELISA results demonstrated that overexpression of IRAK1 could memorably attenuate the reduction of AF on IL-6 and TNF-*α* levels in Ox-LDL-induced HUVECs (Figure 3(b)). Besides, we found that the remarkable increase of cholesterol efflux mediated by high doses of AF could also be weakened by IRAK1 overexpression in Ox-LDL-induced HUVECs (Figure 3(c)). As a result, we testified that IRAK1 was necessary for the inhibition of AF on the inflammation and the promotion on viability and cholesterol efflux in Ox-LDL-induced HUVECs.

### 3.4. IRAK1 Was Involved in AF-Mediated IRAK1-TAK1, Apoptosis, and Mitochondrial Fusion in Ox-LDL-Induced HUVECs

Furthermore, we verified whether overexpression of IRAK1 also could affect AF-mediated IRAK1-TAK1, apoptosis, and mitochondrial fusion in Ox-LDL-induced HUVECs. As denoted in Figure 4(a), the inhibition of p-IRAK1 and p-TAK1 expressions mediated by high doses of AF also could be prominently reversed by IRAK1 overexpression in Ox-LDL-induced HUVECs. Besides, we discovered that overexpression of IRAK1 could notably reverse the downregulation of apoptosis-related proteins (Bax and caspase 3) and the upregulation of mitochondrial fusion-related proteins (MFN1, MFN2, and OPA1), which were mediated by high doses of AF in Ox-LDL-induced HUVECs (Figure 4(b)). Similarly, IF results also indicated that overexpression of IRAK1 could dramatically increase the level of p-TAK1, which has been repressed by high doses of AF in Ox-LDL-induced HUVECs (Figure 4(c)). Overall, we certified that AF could restrain IRAK1-TAK1 and apoptosis and accelerate mitochondrial fusion by downregulating IRAK1 in Ox-LDL-induced HUVECs.

## 4. Discussion

AS is a frequent disease of the cardiocerebrovascular system, the paramount risk factor of which is dyslipidemia [4]. Vascular endothelial cells have been reported to participate in several vascular physiological functions, such as angiogenesis, blood barrier function, vasoconstriction, and relaxation [30, 31]. Dysfunction of vascular endothelium is considered to be the initial link causing AS and is in connection with multiple CVDs [11, 12]. Increased apoptosis of endothelial cells can cause damage to vascular endothelial structure and endothelial cell dysfunction, thus inducing vasculopathy [32]. Abundant researches demonstrated that high fat stress, especially Ox-LDL, can induce endothelial cell functional impairment and mediate the upregulation of cell adhesion molecules, inflammatory chemokines, and other proinflammatory mediators, which is the initial stage of AS [33, 34]. Therefore, the HUVEC injury model induced by Ox-LDL was selected in this study to study the mechanism of AF in the process of AS. AF, as a monoterpene glycoside, is the main component of RPR and RPA [25]. Based on the latest reports, AF could ameliorate pulmonary inflammation mediated ovalbumin in asthmatic mice [22, 23]; AF could alleviate memory deficits through inhibiting mitochondrial dysfunction [24]; AF also could prevent the formation of THP-1-derived foam cells by LOX-1/NF-*κ*B pathway [25]. In our study, we further proved that AF could dramatically facilitate viability and cholesterol efflux and prevent inflammation, oxidative stress, and apoptosis in Ox-LDL-induced HUVECs, indicating that AF has a significant weakening effect on Ox-LDL-induced HUVEC injury.

Mitochondria is a highly dynamic organelle that continuously fuses and divides, which is of great significance for the integrity, quality, and spatial distribution of mitochondria [35]. And MFN1, MFN2, and OPA1 are the key regulatory proteins involved in mitochondrial fusion [36]. MFN1 and MFN2 are responsible for mediating the fusion process of mitochondrial outer membrane [37]. The fusion process of mitochondrial intima is cooperatively completed by MFN1 or MFN2 and OPA1 [38]. Mitochondrial fusion has been reported to be associated with CVD, especially AS [39, 40]. For instance, metformin could inhibit AS through Drp1-mediated mitochondrial fission [41]; resveratrol could weaken HUVEC injury by regulating mitochondrial fusion [42]; Ox-LDL could result in endothelial apoptosis by suppressing mitochondrial fusion [43]. In our study, we further testified that AF could prominently upregulate MFN1, MFN2, and OPA1 in Ox-LDL-induced HUVECs, suggesting that AF could induce mitochondrial fusion in Ox-LDL-induced HUVECs. Therefore, these data provide further evidence that AF can mitigate AS.

IRAK family is a family of protein kinases involved in TLR signal transduction [44]. IRAK1, as a key signal regulator in the IRAK family, also plays an active regulatory role in signal transduction [45]. When the TLR family of receptors are activated, IRAK1 can phosphorylate and interact with TRAF6, which induces the activation and nuclear translocation of NF-*κ*B and further activates the production of vast pro-inflammatory cytokines [46, 47]. And this proinflammatory cascade is crucial to the pathogenesis of AS [48]. Therefore, inhibition of the IRAK1 signaling pathway is valuable to minimize the inflammatory cascade-mediated tissue injury. TAK1, also known as MAP3K7 or MEKK7, is a key signal transduction protein related to multiple processes, such as innate immunity, adaptive immunity, vascular development, and tumor formation [49–51]. TAK1 has also been reported to be activated by TGF-*β*, bone morphogenetic protein (BMP), and a range of inflammatory cytokines [52]. And IRAK-TAK1 pathway has also been certified to be associated with multiple inflammatory diseases [53, 54]. In our study, we first proved that AF could memorably downregulate p-IRAK1 and p-TAK1 in Ox-LDL-induced HUVECs, indicating the inhibitory effect of AF on IRAK1-TAK1 pathway in AS. Above all, we found that overexpression of IRAK1 could reverse the effects of AF on inflammation, apoptosis, viability, cholesterol efflux, and mitochondrial fusion in Ox-LDL-induced HUVECs, suggesting that IRAK1 is crucial in the mitigation of AS mediated by AF.

Finally, our findings show that AF can halt the course of AS by inhibiting apoptosis and inducing mitochondrial fusion via IRAK1. As a result, we hypothesized that AF could be a molecular medication for the treatment of AS.

## Figures and Tables

**Figure 1:** AF memorably induced viability and cholesterol efflux and repressed inflammation, ROS production, and apoptosis in Ox-LDL-induced HUVECs. (a) After 0, 4, 20, 100, 200, and 300 *μ*M of AF stimulation, the toxicity of AF was monitored using CCK-8 in HUVECs by calculating the inhibition rate; ^∗^*P* < 0.05, ∗∗*P* < 0.01, and ^∗∗∗^*P* < 0.001 compared with the 0 *μ*M AF group. (b) After 4 *μ*M AF (AF-L) and 100 *μ*M AF (AF-H) treatment, cell viability was confirmed by CCK-8 in 100 mg/L Ox-LDL-induced HUVECs; ∗*P* < 0.05 compared with the control group and ^#^*P* < 0.05 compared with the Ox-LDL group. (c) Percentage of cholesterol efflux (i.e., the proportion of labelled cholesterol moved from cells to the specified acceptor) was tested using the corresponding kit in Ox-LDL-induced HUVECs after 4 *μ*M AF(AF-L) and 100 *μ*M AF(AF-H) treatment; ^∗^*P* < 0.05 compared with the control group and ^#^*P* < 0.05 compared with the Ox-LDL group. (d) The levels of IL-6 and TNF-*α* were verified by ELISA kits in Ox-LDL-induced HUVECs after AF exposure; ^∗^*P* < 0.05 and ^∗∗^*P* < 0.01 compared with the control group; ^#^*P* < 0.05 and ^##^*P* < 0.01 compared with the Ox-LDL group. (e) The influence of low- and high-dose AF on ROS production was confirmed using flow cytometry in Ox-LDL-induced HUVECs; ^∗^*P* < 0.05 compared with the control group and ^#^P < 0.05 compared with the Ox-LDL group. (f) The impact of AF on cell apoptosis was identified by flow cytometry in Ox-LDL-induced HUVECs; ^∗^*P* < 0.05 compared with the control group and ^#^*P* < 0.05 compared with the Ox-LDL group.

**Figure 2:** AF dramatically suppressed IRAK1-TAK1 and apoptosis and induced mitochondrial fusion in Ox-LDL-induced HUVECs. (a) After 4 *μ*M (AF-L) or 100 *μ*M (AF-H) of AF induction, the levels of p-IRAK1, IRAK1, p-TAK1, and TAK1 were identified through western blotting analysis in 100 mg/L Ox-LDL-stimulated HUVECs. “1” and “2” are representative of three biological repetitions. (b) Western blotting analysis of apoptosis-related proteins (Bax and caspase 3) and mitochondrial fusion-related proteins (MFN1, MFN2, and OPA1) in 100 mg/L Ox-LDL-induced HUVECs after 4 *μ*M AF (AF-L) and 100 *μ*M AF (AF-H) treatment. “1” and “2” are representative of three biological repetitions. (c) The expression and location of p-TAK1 were verified via IF assay in Ox-LDL-induced HUVECs after processing with AF. Magnification, 200×; scale bar = 20 *μ*m.

**Figure 3:** IRAK1 overexpression prominently reversed the influences of AF on viability, inflammation, and cholesterol efflux in Ox-LDL-induced HUVECs. Ox-LDL-treated HUVECs were treated with 100 *μ*M AF or/and IRAK1-overexpressed plasmid, respectively. ^∗^*P* < 0.05, ^∗∗^*P* < 0.01, and ^∗∗∗^*P* < 0.001 compared with the control group; ^#^*P* < 0.05, ^##^*P* < 0.01, and ^###^*P* < 0.001 compared with the Ox-LDL group; ^$^*P* < 0.05, ^$$^*P* < 0.01, and ^$$$^*P* < 0.001 compared with the Ox-LDL+AF-H group. (a) Cell viability was confirmed through CCK-8 in the treated HUVECs. (b) Changes in IL-6 and TNF-*α* levels were monitored by ELISA kits in each group; ∗*P* < 0.05 compared with the control group; ^#^*P* < 0.05 compared with the Ox-LDL+AF-H group; ^$^*P* < 0.05 compared with the control group. (c) Cholesterol efflux was certified with the kit in each group.

**Figure 4:** IRAK1 was required for AF-mediated IRAK1-TAK1, apoptosis, and mitochondrial fusion in Ox-LDL-induced HUVECs. 100 *μ*M AF and IRAK1-overexpressed plasmid were applied to treat Ox-LDL-processed HUVECs, respectively. (a) p-IRAK1, IRAK1, p-TAK1, and TAK1 expressions were certified via western blotting analysis. “1” and “2” are representative of three biological repetitions. (b) Western blotting analysis of apoptosis-related proteins (Bax and caspase 3) and mitochondrial fusion-related proteins (MFN1, MFN2, and OPA1) in the treated HUVECs. “1” and “2” are representative of three biological repetitions. (c) The expression and location of p-TAK1 was determined using IF assay in the treated HUVECs. Magnification, 200×; scale bar = 20 *μ*m.

## Data Availability

The data utilized which corroborated this study's conclusions are accessible once requested from the corresponding author.
